# Risky decision-making and delusion proneness: An initial examination

**DOI:** 10.1016/j.heliyon.2019.e02767

**Published:** 2019-11-14

**Authors:** Meisha Runyon, Melissa T. Buelow

**Affiliations:** The Ohio State University Newark, 1179 University Drive, Newark, OH, 43055, USA

**Keywords:** Psychology, Jumping to conclusions, Iowa gambling task, Risky decision making, Game of dice task, Delusion proneness

## Abstract

Delusion proneness is an individual-differences characteristic, existing on a continuum from no delusional thoughts to a diagnosis of schizophrenia. Previous research found individuals high in delusion proneness request less information to make decisions, potentially making a decision without sufficient information (jumping to conclusions). The present study examined risky decision-making as a function of delusion proneness. Participants (*n* = 102) completed the Peters Delusions Inventory to assess delusion proneness, and the Iowa Gambling Task (IGT) and Game of Dice Task (GDT) to assess risky decision-making. Although no significant results emerged on the GDT, those scoring higher in delusion proneness decided more advantageously on the IGT than those scoring lower in delusion proneness. Exploratory analyses indicated no significant relationship between gender and task performance. The present study provides further insight into risky decision making as a function of delusion proneness.

## 1 Introduction

Decision-making deficits are seen across a variety of diagnosable mental health conditions, as well as in the general population as a function of individual differences factors such as impulsivity. Utilizing behavioral decision-making tasks, multiple studies found impairments among individuals with a diagnosis of schizophrenia compared to healthy controls (Bark et al., 2005; Brown et al., 2015; Caletti et al., 2013; Cheng et al., 2012; Fond et al., 2013; Hori et al., 2014; Premkumar et al., 2008; Wasserman et al., 2012; Yip et al., 2009). Delusional beliefs—imprecise thoughts that exist despite evidence to the contrary (Peters et al., 1999)—are thought to exist on a spectrum, where delusions strong enough to be associated with psychotic disorders are at one extreme and the absence of delusions at the other extreme (So and Kwok, 2015). Existing between the two ends of this spectrum is delusion proneness, an individual-differences characteristic focused on the frequency and type of delusional beliefs (Peters et al., 1999). Individuals high in delusion proneness vary in frequency of the delusions, in turn leading to differing effects on the individual's life and potentially on decision-making tasks. Delusions are multidimensional, with three characteristics of particular interest: conviction (strength of the belief), preoccupation (amount of time spent on the belief), and distress (effect on daily life) (Peters et al., 1999). Levels of conviction, preoccupation, and distress can vary for each individual, just as frequency of the delusional belief varies.

Previous research suggests that individuals across the delusional belief spectrum, including those who are delusion-prone and those with a diagnosis of schizophrenia, show a “jumping to conclusions” (JTC) bias (Linney et al., 1998). The JTC bias is evident when individuals request less information prior to making a decision, leading to a less advantageous decision than those requesting more information. Those with a diagnosis of schizophrenia (Klein and Pinkham, 2018) and those high in delusion proneness (Dudley et al., 1997; Fine et al., 2007; Garety and Freeman, 2013; Linney et al., 1998; Moritz et al., 2016; So and Kwok, 2015; van der Leer et al., 2015; van der Leer and McKay, 2014) show a JTC bias compared to healthy controls. It is possible that this bias could negatively affect decisions across different behavioral decision-making tasks, such as the Iowa Gambling Task (IGT; Bechara et al., 1994). On the IGT, participants must sample from each deck of cards in order to learn the relative risks and benefits associated with each deck. Failing to adequately sample from each deck could lead to worse outcomes. On the Game of Dice Task (GDT; Brand et al., 2005), however, participants are explicitly given information about the risks and benefits of their decisions at the start of the task, and performance on this task might better inform our understanding of the JTC bias. Specifically, the IGT, at least in the early trials, is thought to assess decision making under ambiguity, as participants must sample from each deck to learn the relative risks and benefits associated with each. The GDT, on the other hand, assesses risky decision making when the risks and benefits of each selection are explicitly stated at the start of the task. Utilizing these two measures in the same study could help our understanding of whether poor performance on decision making tasks as a function of delusion proneness is due to an information sampling impairment or a decision making impairment.

The present study examines risky decision-making as a function of delusion proneness. Just as individuals with high levels of trait impulsivity but not a diagnosis of Attention-Deficit/Hyperactivity Disorder (ADHD) show riskier decisions than those low on trait impulsivity (e.g., Buelow and Suhr, 2013; Burdick et al., 2013; Franken and Muris, 2005; Sweitzer et al., 2008), it is possible that those high in delusion proneness but without a diagnosis of schizophrenia may also show riskier decisions than those low in delusion proneness. Assessing the tendency of those across the spectrum of delusional thought processes to engage in risky decision making is important to our understanding of how decision making can be affected by state and trait processes. If delusion proneness is a precursor to schizophrenia and decision making impairments are found, then this would provide evidence that the decision making impairments seen in schizophrenia could predate full development of the symptoms. In the present study, it was hypothesized that individuals high in delusion proneness will be riskier on the IGT and GDT than individuals low in delusion proneness. As a secondary aim, relationships between risky decision making and levels of conviction, preoccupation, and distress associated with the delusional beliefs were examined.

## 2 Methods

### 2.1 Participants

An a priori power analysis was conducted to determine the required sample size to determine a medium effect for α = .05 and power = .80. The power analysis indicated a total sample of 82 participants was needed for adequate power in the correlational analyses, and samples of 46–128 for between-group comparisons. Participants were 102 undergraduate student participants, ages 18–23 (*M*_age_ = 18.55, *SD*_age_ = 0.89), at a regional campus of a large Midwestern university. Thirty-four self-reported their gender as male and 64.6% self-reported their ethnicity as Caucasian. All participants received course credit for their participation.

### 2.2 Measures and procedure

The university's Institutional Review Board approved the present study, and participants provided informed consent. Participants completed the 40-item Peters Delusion Inventory (PDI; Peters et al., 1999) to assess level of delusion proneness. Participants respond to a series of questions indicating: 1) level of agreement with the question (yes [*1*] or no [*0*]), and 2) level of conviction, preoccupation, and distress (1 [*not at all*] to 5 [*very*] scale). An overall level of delusion proneness was calculated from the yes/no responses (range: 0–40; *M* = 10.11, *SD* = 7.22). Average scores were calculated for conviction, preoccupation, and distress, with higher average scores indicating higher levels of these factors.

Next, participants completed the GDT and IGT to assess risky decision-making. On the GDT (Brand et al., 2005), participants are asked to maximize their profit by rolling a virtual die 18 times. Before each roll, participants predict the die roll by choosing a single number or combination of up to four numbers. Making a selection of a single number carries a risk of $1000, two numbers is $500, three numbers is $200, and four numbers is $100. Selecting three or four numbers is considered a safe decision, whereas selecting one or two numbers is considered a risky decision (Brand et al., 2005). This information is made available to participants at the start of the task (i.e., did not depend on decision feedback during the task). For the present study, a net score was calculated by subtracting the number of risky selections from the number of safe selections (positive scores indicate less risky decision-making).

The standard computerized IGT was also administered (Bechara, 2007). Participants are tasked with maximizing their profit over 100 selections from Decks A, B, C, and D. After each selection, participants win money, but sometimes also lose money. Unbeknownst to the participants, and learned through trial-and-error feedback, the decks have varying levels of risk attached to them. Decks A and B produce an average profit of $100 on each selection (high immediate gain), but after 10 selections, have incurred a net loss of $250 (long-term negative consequence). Decks C and D produce an average profit of $50 on each selection (low immediate gain), but after 10 selections, have instead incurred a net gain of $250 (long-term positive consequence). Based on these long-term outcomes, Decks A and B are termed disadvantageous, and continued selection from them indicative of risky decision-making. Decks C and D, on the other hand, are termed advantageous decks. Early selections on the IGT, generally the first 40 trials, are considered decision-making under ambiguity, as participants have not learned the relative risks and benefits of each deck. However, after those 40 trials, the remaining trials are considered decision-making under risk (Brand et al., 2007). For the present study, the number of disadvantageous (A, B) selections was subtracted from the number of advantageous (C, D) selections across the early (Trials 1–40) and later (Trials 41–100) selections. More positive values indicate less risky decision-making.

Participants also reported basic demographic information prior to the debriefing.

### 2.3 Data analysis

Of note, nine participants were missing data on the IGT due to computer malfunction. Thus, the IGT analyses were conducted on a sample of 93 participants and the GDT analyses on a sample of 102 participants. To assess the first hypothesis, two analyses were conducted. First, Pearson's correlations were conducted between PDI total score and performance on the IGT and GDT. Due to mild variations from normality in the IGT and GDT data, nonparametric statistics were used. For the IGT data, the Friedman test was conducted separately among those scoring below the PDI median and those scoring above the PDI median (per the scoring criteria from Peters et al., 1999). For the GDT data, the Mann-Whitney U test was used to assess this variable. To assess the second study aim, correlations were also calculated between levels of conviction, preoccupation, and distress and task performance.

## 3 Results

No significant relationships were found between delusion proneness total score and performance on the GDT or either the earlier or later trials on the IGT (see Table 1; see Figs. 1, 2, and 3 for histograms of the PDI, IGT, and GDT scores and Figs. 4 and 5 for scatterplots). With regard to conviction, distress, and preoccupation, none of these factors was associated with performance on the GDT or IGT.

**Table 1:** Means (*M*), standard deviations (*SD*), and correlations for study variables.

Variable	*M(SD)*	Range	1	2	3	4	5	6	7
PDI-t	10.11 (7.22)	0–29	--	.288**	.342***	.279**	.171	.136	-.141
PDI-d	2.39 (0.95)	1–5		--	.757***	.644***	.075	-.001	-.131
PDI-p	2.50 (0.91)	1–5			--	.910***	.165	.039	-.117
PDI-c	2.58 (0.93)	1–5				--	.129	-.025	-.114
IGT-1	-3.01 (9.61)	-36–40					--	.486***	.196^a^
IGT-2	5.73 (20.81)	-54–60						--	.303**
GDT	4.36 (10.19)	-18–18							--

*p < .05; **p < .01; ***p < .001; ^a^*p* = .06.

*Note*: PDI = Peters Delusion Inventory (t = total score, c = conviction, d = distress; p = preoccupation); IGT = Iowa Gambling Task, advantageous minus disadvantageous selections on early (1) and later (2) trials; GDT = Game of Dice Task, advantageous minus disadvantageous selections.

**Fig. 1:** Histogram of the Peters Delusion Inventory.

**Fig. 2:** Histogram of the Iowa Gambling Task.

**Fig. 3:** Histogram of the Game of Dice Task.

**Fig. 4:** Scatterplot of the Iowa Gambling Task by PDI Score.

**Fig. 5:** Scatterplot of the Game of Dice Task by PDI Score.

Next, the median split was calculated based on a median score of 9.5. Delusion proneness was recoded as 1 (*below median*) and 2 (*above median*). Among those scoring below the PDI median, the Friedman test indicated no significant changes in IGT performance across block, χ^2^(1) = 1.80, *p* = .180. For those scoring above the PDI median, the Friedman test instead indicated more advantageous decisions during the later compared to earlier trials, χ^2^(1) = 8.395, *p* = .004. No significant differences emerged between groups on the GDT, *U =* 1249.50, *p* = .732.

To assess for potential differences in task performance by self-reported gender, due to known differences on the IGT and other tasks (e.g., Businelle et al., 2008; Davis et al., 2007; van den Bos2013), a series of exploratory analyses were conducted. For the GDT data, a permutation test (with gender labels varied in a bootstrap procedure [1000 permutations]) found no significant effect of gender on task performance, *t* = 0.91, *p* = .362. Self-reported gender was also not associated with selections on the early IGT trials, *t* = -1.55, *p* = .123, nor on the later IGT trials, *t* = -0.49, *p* = .624.

## 4 Discussion

The present pilot study examined the potential relationship between delusion proneness, an individual-differences variable, and performance on two common behavioral decision-making tasks, the IGT and GDT. Limited support was found for the hypothesis that participants scoring higher in delusion proneness would be riskier on the tasks than individuals scoring lower in delusion proneness. No overall correlation was found between score on the PDI and task performance, but participants scoring below the median split were riskier on the IGT but not the GDT than participants scoring above it. These results are contrary to previous research examining IGT and GDT performance among individuals with a diagnosis of schizophrenia (Bark et al., 2005; Brown et al., 2015; Cheng et al., 2012), and run counter to previous studies showing a JTC bias as a function of delusion proneness (Linney et al., 1998; So and Kwok, 2015; van der Leer et al., 2015; van der Leer and McKay, 2014). However, to our knowledge this is the first examination of a potential relationship between delusion proneness and performance on either the IGT or GDT. As such, our results should be further investigated in a larger, more diverse sample with a greater range of delusion proneness on the PDI and the distress, preoccupation, and conviction subscales.

Our finding that participants scoring higher in delusion proneness actually used a more advantageous decision-making strategy on the IGT compared to those low in delusion proneness is consistent with some previous research suggesting better task performance among those high in delusion proneness (Freeman et al., 2010; Warman et al., 2007). It is possible that individuals adjust their data gathering abilities to the type of task at hand, expending greater cognitive resources on harder than on easier tasks. The IGT might have been viewed as a harder task, given the limited information made available at the start of the task, and thus the additional expenditure of cognitive resources led to improved performance on the task. It is also possible that participants high in delusion proneness had a higher level of imagination or creativity that resulted in greater strategy use to learn to decide advantageously on the IGT. Finally, it is also possible that individuals high in delusion proneness experience a bias in their ability to use reinforcement-based feedback to learn to decide advantageously. Participants may respond differently to immediate gains versus immediate losses, in turn affecting future decision making strategies on tasks in which participants must learn from feedback such as the IGT. Additional research is needed to replicate and further examine the causes of this unanticipated finding.

The present study is not without limitations. This was a small pilot study focused on undergraduate student participants. Although we were adequately powered to detect medium effects, our results indicated that several effects were likely small. Our group difference on the IGT in particular represented a small effect size, potentially limiting implications of this finding. Future research should utilize larger samples and incorporate cognitive modeling components (e.g., Horstmann et al., 2012; Worthy et al., 2013) to further tease apart the processes affecting decision making on the IGT. It is possible that the full spectrum of the delusion proneness characteristic was not evidenced in this sample, and a follow-up study with a larger, more diverse sample is suggested. It is also possible that the present results were affected by the speed-accuracy trade-off, in that participants slowed down their decision-making processes to arrive at the “correct” or most advantageous decision. This process might in turn have equalized performance across levels of delusion proneness; however, data on decision-making speed was not collected for all participants, making this analysis difficult in our small sample. We also did not collect data on concurrent substance use or mental health diagnoses, which could affect performance on the decision making tasks and should be investigated in future studies.

The present study serves as an initial examination of potential relationships between delusion proneness and performance on behavioral decision-making tasks. Results indicated few relationships between this individual-differences variable and performance on the IGT or GDT, but this might have been affected by characteristics of our study sample. Future research should continue to examine the potential JTC bias as a function of delusion proneness on other decision-making tasks. Future research utilizing both easy and hard tasks in the same study will help elucidate this data gathering deficit in delusion proneness.

## Declarations

### Author contribution statement

M. Buelow: Conceived and designed the experiments; Analyzed and interpreted the data; Contributed reagents, materials, analysis tools or data; Wrote the paper.

M. Runyon: Conceived and designed the experiments; Performed the experiments; Analyzed and interpreted the data; Contributed reagents, materials, analysis tools or data; Wrote the paper.

### Funding statement

This research did not receive any specific grant from funding agencies in the public, commercial, or not-for-profit sectors.

### Competing interest statement

The authors declare no conflict of interest.

### Additional information

Data associated with this study has been deposited at OSF: DOI 10.17605/OSF.IO/C6KXQ.

## References

[bib1] Bark R., Dieckmann S., Bogerts B., Northoff G. (2005). Deficit in decision-making in catatonic schizophrenia: an exploratory study. Psychiatry Res..

[bib2] Bechara A. (2007). Iowa Gambling Task Professional Manual.

[bib3] Bechara A., Damasio A.R., Damasio H., Anderson S.W. (1994). Insensitivity to future consequences following damage to human prefrontal cortex. Cognition.

[bib4] Brand M., Kalbe E., Labudda K., Fujiwara E., Kessler J., Markowitsch H.J. (2005). Decision-making impairments in patients with pathological gambling. Psychiatry Res..

[bib5] Brand M., Recknor E.C., Grabenhorst F., Bechara A. (2007). Decisions under ambiguity and decisions under risk: correlations with executive functions and comparisons of two different gambling tasks with implicit and explicit rules. J. Clin. Exp. Neuropsychol..

[bib6] Brown E.C., Hack S.M., Gold J.M., Carpenter W.T., Fischer B.A. (2015). Integrating frequency and magnitude information in decision-making in schizophrenia: an account of patient performance on the Iowa gambling task. J. Psychiatr. Res..

[bib7] Buelow M.T., Suhr J.A. (2013). Personality characteristics and state mood influence individual deck selections on the Iowa gambling task. Personal. Individ. Differ..

[bib8] Burdick J.D., Roy A.L., Raver C.C. (2013). Evaluating the Iowa gambling task as a direct assessment of impulsivity with low-income children. Personal. Individ. Differ..

[bib9] Businelle M.S., Apperson M.R., Kendzor D.E., Terlecki M.A., Copeland A.L. (2008). The relative impact of nicotine dependence, other substance dependence, and gender on Bechara gambling task performance. Exp. Clin. Psychopharmacol.

[bib10] Caletti E., Paoli R.A., Fiorentini A., Cigliobianco M., Zugno E., Altamura A.C. (2013). Neuropsychology, social cognition, and global functioning among bipolar, schizophrenic patients and healthy controls: preliminary data. Front. Hum. Neurosci..

[bib11] Cheng G.F., Tang J.Y., Li F.S., Lau E.Y., Lee T.C. (2012). Schizophrenia and risk-taking: impaired reward but preserved punishment processing. Schizophr. Res..

[bib12] Davis C., Patte K., Tweed S., Curtis C. (2007). Personality traits associated with decision making deficits. Personal. Individ. Differ..

[bib13] Dudley R.E., John C.H., Young A.W., Over D.E. (1997). Normal and abnormal reasoning in people with delusions. Br. J. Clin. Psychol..

[bib14] Fine C., Gardner M., Craigie J., Gold I. (2007). Hopping, skipping or jumping to conclusions? Clarifying the role of the JTC bias in delusions. Cogn. Neuropsychiatry.

[bib15] Fond G., Bayard S., Capdevielle D., Del-Monte J., Mimoun N., Raffard S. (2013). A further evaluation of decision-making under risk and under ambiguity in schizophrenia. Eur. Arch. Psychiatry Clin. Neurosci..

[bib16] Franken I.H.A., Muris P. (2005). Individual differences in decision-making. Personal. Individ. Differ..

[bib17] Freeman D., Pugh K., Vorontsova N., Antley A., Slater M. (2010). Testing the continuum of delusional beliefs: an experimental study using virtual reality. J. Abnorm. Psychol..

[bib18] Garety P.A., Freeman D. (2013). The past and future of delusions research: from the inexplicable to the treatable. Br. J. Psychiatry.

[bib19] Hori H., Yoshimura R., Katsuki A., Atake K., Nakamura J. (2014). Relationships between brain-derived neurotrophic factor, clinical symptoms, and decision-making in chronic schizophrenia: data from the Iowa gambling task. Front. Behav. Neurosci..

[bib20] Horstmann A., Villringer A., Neumann J. (2012). Iowa gambling task: there is more to consider than long-term outcome. Using a linear equation model to disentangle the impact of outcome and frequency of gains and losses. Front. Neurosci..

[bib21] Klein H.S., Pinkham A.E. (2018). Examining reasoning biases in schizophrenia using a modified “jumping to conclusions” probabilistic reasoning task. Psychiatry Res..

[bib22] Linney Y.M., Peters E.R., Ayton P. (1998). Reasoning biases in delusion-prone individuals. Br. J. Clin. Psychol..

[bib23] Moritz S., Scheu F., Andreou C., Pfueller U., Weisbrod M., Roesch-Ely D. (2016). Reasoning in psychosis: risky but not necessarily hasty. Cogn. Neuropsychiatry.

[bib24] Peters E.R., Joseph S.A., Garety P.A. (1999). Measurement of delusional ideation in the normal population: introducing the PDI (Peters et al. delusions inventory). Schizophr. Bull..

[bib26] Premkumar P., Fannon D., Kuipers E., Simmons A., Frangou S., Kumari V. (2008). Emotional decision-making and its dissociable components in schizophrenia and schizoaffective disorder: a behavioural and MRI investigation. Neuropsychologia.

[bib27] So S.H., Kwok N.T. (2015). Jumping to conclusions style along the continuum of delusions: delusion-prone individuals are not hastier in decision-making than healthy individuals. PLoS One.

[bib28] Sweitzer M.M., Allen P.A., Kaut K.P. (2008). Relation of individual differences in impulsivity to nonclinical emotional decision making. J. Int. Neuropsychol. Soc..

[bib29] van den Bos R., Homberg J., de Visser L. (2013). A critical review of sex differences in decision-making tasks: focus on the Iowa gambling task. Behav. Brain Res..

[bib30] van der Leer L., Hartig B., Goldmanis M., McKay R. (2015). Delusion proneness and ‘jumping to conclusions’: relative and absolute effects. Psychol. Med..

[bib31] van der Leer L., McKay R. (2014). “Jumping to conclusions” in delusion-prone participants: an experimental economics approach. Cogn. Neuropsychiatry.

[bib32] Warman D.M., Lysaker P.H., Martin J.M., Davis L., Haudenschield S.L. (2007). Jumping to conclusions and the continuum of delusional beliefs. Behav. Res. Ther..

[bib33] Wasserman J.I., Barry R.J., Bradford L., Delva N.J., Beninger R.J. (2012). Probabilistic classification and gambling in patients with schizophrenia receiving medication: comparison of risperidone, olanzapine, clozapine and typical antipsychotics. Psychopharmacology.

[bib34] Worthy D.A., Hawthorne M.J., Otto A.R. (2013). Heterogeneity of strategy use in the Iowa gambling task: a comparison of win-stay/lose-shift and reinforcement learning models. Psychon. Bull. Rev..

[bib35] Yip S.W., Sacco K.A., George T.P., Potenza M.N. (2009). Risk/reward decision-making in schizophrenia: a preliminary examination of the influence of tobacco smoking and relationship to Wisconsin card sorting task performance. Schizophr. Res..

